# High-Fat Diet Increases Bone Loss by Inducing Ferroptosis in Osteoblasts

**DOI:** 10.1155/2022/9359429

**Published:** 2022-10-14

**Authors:** RunJiu Zhu, ZhaoFu Wang, Yuan Xu, HaoYang Wan, Xin Zhang, MingRui Song, Hong Yang, Yu Chai, Bin Yu

**Affiliations:** ^1^Division of Orthopaedic Surgery, Department of Orthopaedics, Nanfang Hospital, Southern Medical University, Guangzhou 510515, China; ^2^Guangdong Provincial Key Laboratory of Bone and Cartilage Regenerative Medicine, Nanfang Hospital, Southern Medical University, Guangzhou 510515, China; ^3^Department of Orthopaedics, People's Hospital of Ningxia Hui Autonomous Region, Yinchuan 750000, China; ^4^Department of Orthopaedics & Traumatology, Wuyi Hospital of Traditional Chinese Medicine, Jiangmen 523000, China; ^5^Department of Respiratory and Critical Care Medicine, Nanfang Hospital, Southern Medical University, Guangzhou 510515, China

## Abstract

Current research suggests that chronic high-fat dietary intake can lead to bone loss in adults; however, the mechanism by which high-fat diets affect the development of osteoporosis in individuals is unclear. As high-fat diets are strongly associated with ferroptosis, whether ferroptosis mediates high-fat diet-induced bone loss was the focus of our current study. By dividing the mice into a high-fat diet group, a high-fat diet + ferroptosis inhibitor group and a normal chow group, mice in the high-fat group were given a high-fat diet for 12 weeks. The mice in the high-fat diet + ferroptosis inhibitor group were given 1 mg/kg Fer-1 per day intraperitoneally at the start of the high-fat diet. Microscopic CT scans, histological tests, and biochemical indicators of ferroptosis were performed on bone tissue from all three groups at the end of the modelling period. Mc3t3-E1 cells were also used in vitro and divided into three groups: high-fat medium group, high-fat medium+ferroptosis inhibitor group, and control group. After 24 hours of incubation in high-fat medium, Mc3t3-E1 cells were assayed for ferroptosis marker proteins and biochemical parameters, and osteogenesis induction was performed simultaneously. Cellular alkaline phosphatase content and expression of osteogenesis-related proteins were measured at day 7 of osteogenesis induction. The results showed that a high-fat diet led to the development of femoral bone loss in mice and that this process could be inhibited by ferroptosis inhibitors. The high-fat diet mainly affected the number of osteoblasts produced in the bone marrow cavity. The high-fat environment in vitro inhibited osteoblast proliferation and osteogenic differentiation, and significant changes in ferroptosis-related biochemical parameters were observed. These findings have implications for the future clinical treatment of bone loss caused by high-fat diets.

## 1. Introduction

Overweight and obesity are not only significant risk factors for cardiovascular disease, hypertension, and other cardiovascular diseases [1, 2] but also have adverse effects on bone through various mechanisms such as affecting bone formation and the bone marrow microenvironment [3]. The diseases arising from abnormal lipid metabolism and the development of osteoporosis are currently receiving increasing attention from researchers, who have found that patients with hyperlipidaemia can experience both bone loss and osteoporosis [4, 5]. At the same time, patients who develop osteoporosis and reduced bone mass also have abnormal lipid metabolism and vascular calcification [6], suggesting that osteoporosis and lipid metabolism may be causally linked. Osteoporosis is a systemic skeletal disease characterized by a reduction in bone mineral density and bone strength, which increases the risk of fracture due to increased bone fragility [7]. The pathogenesis of osteoporosis is mainly due to a disruption of the balance between bone resorption and bone formation, resulting in a disorder of bone metabolism, which is associated with a decrease in the number and function of osteoblasts [8, 9]. The process of bone reconstruction is based on a dynamic balance between the two main mechanisms of osteoclast-associated bone resorption and osteoblast-associated bone formation [8]. And osteoblast cell death is an important pathogenic mechanism in osteoporosis [9]. Cell death is caused by a variety of mechanisms. The modes of cell death include autophagy, pyroptosis, senescence, and ferroptosis [10–12]. Osteoporosis is currently well studied in cellular senescence [13], cellular autophagy [14], and cellular pyroptosis [15], but less studied in cellular ferroptosis. Iron overload has been reported in the literature to cause osteoporosis [16, 17]. Therefore, controlling ferroptosis could be effective in preventing osteoporosis or promoting osteoblast osteogenic capacity. We therefore shifted our experimental focus to investigate the phenomenon of bone loss triggered by ferroptosis in osteoblasts. Ferroptosis was first proposed by Dixon et al. in 2012 [18] and is essentially the result of lipid peroxidation and excessive accumulation of intracellular reactive oxygen species due to damage to the cellular antioxidant system, which in turn leads to ferroptosis [19]. In ferroptosis, inhibition of glutathione peroxidase 4 and cystine/glutamate antiporter protein affects cysteine metabolism and promotes lipid peroxidation in cells [20]. Excess intracellular divalent iron causes ferroptosis in cells through the Fenton reaction [18]. In recent years, researchers have found that cells in high-fat environments are prone to ferroptosis [21, 22]. Ferroptosis plays an important role in cardiovascular diseases caused by high-fat diets [23, 24]. Therefore, it is reasonable to speculate that ferroptosis in osteoblasts in a high-fat environment is an important pathway for bone loss due to high-fat diets when mice are given a long-term high-fat diet. This holds great promise for the future clinical treatment of osteoporosis caused by high-fat diets.

## 2. Materials and Methods

### 2.1. Animals

The experimental protocol was approved by the Southern Hospital Animal Care and Use Committee and was conducted in accordance with the Southern Hospital Southern Medical University Guide for Laboratory Animals. The experimental mice were housed in a conventional experimental environment where the mice underwent a 12-hour light/12-hour dark cycle daily and were kept at a controlled temperature of around 25°C and 50% relative humidity with free access to food and drinking water. After one week of adaptive feeding, the mice were randomly assigned to three groups: normal control mice, high-fat diet mice, and high-fat diet + inhibitor mice. Mice in the high-fat diet group and mice in the high-fat diet + Fer-1 group were given HFD (D12492, Research Diet, USA) for a total of 12 weeks at the time of moulding. Mice in the high-fat diet + Fer-1 group were given a high-fat diet along with an intraperitoneal injection of 1 mg/kg Fer-1 (MCE, HY-100579, USA) starting daily. After the end of moulding, the mice were executed by the cervical dislocation method, and tissues were extracted for further experiments.

### 2.2. Micro-CT

After execution of the mice, the leg tissue was cut, and the femur was removed and washed in saline. This was followed by overnight fixation in 4% paraformaldehyde in a cold room at 4°C and studied using high-resolution CT scans (Skyscan 1172, Bruker MicroCT, Kontich, Belgium). The scans were performed using an X-ray energy of 55 kVp and a current of 145 mA, with a voxel size of 12 *μ*m and an integration time of 400 ms. To get a clear picture of the changes in trabeculae in the region of the femoral epiphysis in mice, we used quantitative analysis which was performed using IPL software (Image Processing Language V5.15, Scanco Medical AG, Switzerland) for quantitative analysis. The region of the experiment (ROI) was selected starting 1 mm below the reference level of the distal epiphyseal plate and extending 2 mm in length in a distal direction for histomorphometric analysis of the trabeculae.

### 2.3. Histochemistry Staining

The femurs of the mice were separated from the soft tissue and fixed in 4% paraformaldehyde for 36 hours. This was followed by decalcification in 0.5 M ethylenediaminetetraacetic acid (EDTA, pH 8.0) for 10 days, followed by paraffin embedding. The resulting paraffin-embedded samples were cut longitudinally into 4 *μ*m-thick sections. Alkaline phosphatase (ALP) staining and antitartrate acid phosphatase (TRAP) staining were performed, together with eosin (H&E) staining to visualize the histomorphology. To better assess the number of osteoblasts and osteoclast activity on the surface of bone trabeculae in experimental mice, the Wako TRAP/ALP stain kit (Cat. 294-67001) was used, and the manufacturer's instructions were followed: number of osteoblasts per millimeter of bone surface (N. of Ob/mm) and number of TRAP+ cells per millimeter of bone surface (N. of TRAP+). The number of osteoblasts per millimeter of bone surface (N. of Ob/mm) and the number of TRAP+ cells per millimeter of bone (N. of TRAP+/mm) were quantified.

### 2.4. Immunofluorescence Staining of Tissues and Cells

#### 2.4.1. Immunofluorescence Staining of Tissues

The 4 *μ*m paraffin wax was dewaxed and rehydrated into sodium citrate antigen repair solution and water bathed for 2 hours at 75°C, rinsed with PBS 3 times/min, and closed with BSA for one hour. This was followed by incubation with primary antibody GPX4 (Abcam, ab125066, 1 : 200) overnight at 4°C and then with fluorescently labelled secondary antibody for 1 hour at room temperature. Tissues were stained with anti-fluorescence-attenuated blocker containing DAPI as a counterstain (S2110, Solarbio, China). Sections were viewed with a Zeiss Axio Imager.D2 (Axio imager M2 Microscope, Germany). We randomly selected two nonoverlapping positions in three sections of each mouse specimen to quantify positive cells.

#### 2.4.2. Immunofluorescence Staining of Cells

Cells were removed from the cell incubator after 24 hours of high-fat medium stimulation and Mc3t3-E1-E1 cells that had undergone seven days of osteogenic differentiation after high-fat medium stimulation, washed three times with PBS, and then, fixed with 4% paraformaldehyde for 15 minutes before washing the cells three times with PBS. The membrane was broken with 0.1% TritonX-100 for 15 minutes, followed by closure with 5% BSA for one hour. At the end of the closure high-fat medium was used to stimulate the cells for 24 hours after stimulation with primary antibodies Gpx4 (Abcam, ab125066, 1 : 50), Slc7a11 (Proteintech, 26864-1-AP, 1 : 50), and Ki67 (Abcam, ab15580, 1 : 50) to observe intracellular ferroptosis marker proteins and proliferation of changes. Cells undergoing seven-day osteogenic differentiation were treated with primary antibodies Osterix (Abcam, ab209484,1 : 50), Osteocalcin (Proteintech, 23418-1-AP, 1 : 50), and Rux2 (HUABIO, ET1612-47, 1 : 50) to observe changes in intracellular osteogenic-associated proteins. Cells were observed with a Zeiss Axio Imager.D2 (Axio imager M2 microscope, Germany).

### 2.5. Biochemical Analysis

The levels of reduced GSH/GSSG, total GSH (G263, Tong Ren, Japan), malondialdehyde (M496, Tong Ren, Japan), and divalent iron ions (l291, Tong Ren, Japan) in mouse bone tissue and Mc3t3-E1 cells were measured using commercial kits according to the manufacturer's instructions. Measurements were made using commercial kits, following the manufacturer's instructions.

### 2.6. Cell Culture

MC3T3-E1 (GNM15, Cell Bank of Typical Culture Preservation Committee of Chinese Academy of Sciences, China) cells were cultured in medium containing 10% FBS in *α*-MEM. To investigate whether osteoblasts under high-fat condition media (Pythonbio, AAPR156-D500, China) undergo ferroptosis and have reduced osteogenic capacity, we seeded MC3T3-E1 cells at a density of 1 × 10^5^ cells/well on six-well plates. Cells were divided into control, high-fat, and high-fat plus Ferrostatin-1 groups at a concentration of 5 *μ*mol/l. Cells were collected 24 h later for ferroptosis-related assays. For osteogenic differentiation, MC3T3-E1 cells were divided into control group, high-fat group, and high-fat plus Ferrostatin-1 group with Ferrostatin-1 (MCE, HY-100579, China) at a concentration of 5 *μ*mol/l. After 24 hours of treatment in the high-fat and high-fat + Ferrostatin-1 groups, the medium was changed back to the conventional osteogenic differentiation induction medium. On the seventh day, ALP staining and immunofluorescence staining for bone-formation-associated proteins were performed, and the results of ALP staining were quantified.

### 2.7. Osteogenic Differentiation of Cells and ALP Staining

Alkaline phosphatase (ALP) staining assays were used to assess the effect of inhibition of cellular ferroptosis under high-lipid conditions on osteogenic differentiation of Mc3t3-E1cells. Mc3t3-E1 cell suspensions were added to 24-well plates (2 × 10^4^ cells per well) and incubated in a conventional incubator for 12 hours. The medium was then changed to regular medium, high-fat medium, and high-fat plus Ferrostatin-1 medium. After 24 hours of incubation, all media were changed to osteogenic differentiation induction medium, which was prepared with 50 *μ*g/ml ascorbic acid (Sigma, A4544-25G), 10 nmol/l dexamethasone (MCE, HY-14648), and 10 mmol/l *β*-glycerophosphate (Sigma, G9422-10G). Seven days after osteogenic induction, half of the cells were stained for ALP using the ALP staining kit for the plates (Beyotime, C3206), and staining was performed according to the kit guidelines. Observation was made with a bright-field microscope. Photographs were then taken with a bright-field microscope ((OLYMPUS, BX63). The other half was assayed for ALP activity using the ALP quantification kit. The supernatant was collected, and the absorbance was measured at 405 nm (Beyotime, P0321S), and the cellular ALP activity was counted quantitatively.

### 2.8. Statistics

All quantitative data were expressed as mean ± S.E.M. For cell culture experiments, all results were obtained from independent replicates of the experiments, which were repeated independently at least three times. For comparisons between two groups, independent Student's *t*-tests were used. One-way analysis of variance (ANOVA) and Bonferroni post hoc tests were used for multiple comparisons. Statistical analysis software was used for the data using GraphPad, version 7.0 software (GraphPad Software, USA). *P* values < 0.05 considered to be a statistically significant difference.

## 3. Results

### 3.1. Ferroptosis Inhibitor Ferrostatin-1 Can Prevent HFD-Induced Bone Loss

To research the efficacy of Ferrostatin-1 on bone formation and bone resorption in high-fat diet mice, we used a model of bone loss induced by a long-term high-fat diet. Mice fed a high-fat diet were given intraperitoneal injections of Ferrostatin-1, and the results showed that the administration of a high-fat diet to mice resulted in a reduction in femoral trabecular bone mass. This high-fat diet-mediated bone loss was inhibited by Ferrostatin-1. Morphometric analysis of the distal femur showed that BV/TV and number (Tb.N) were reduced and that this change was inhibited by Ferrostatin-1. However, the effect of Ferrostatin-1 on trabecular bone thickness (Tb.Th) but trabecular bone separation (Tb.Sp) in mice on a high-fat diet was not statistically significant (Figure 1(d)).

### 3.2. High-Fat Diet Induces Loss of Osteoblasts

As a result of the analysis of micro-CT data, a chronic high-fat diet alters the bone structure of long bones in mice. We investigated in our experiments whether the bone marrow microenvironment of HFD-fed mice leads to a decrease in the number of osteoblasts. It was again verified by histological examination of HE staining that bone loss in high-fat diet mice could be mitigated by Ferrostatin-1, as shown by H&E staining (Figure 2(a)). During the course of our study, we identified an important role for the precursors of osteoblast formation. Proosteoblasts are an important population for bone formation in the bone marrow cavity. In order to detect changes in osteoblasts on the surface of bone trabeculae. ALP staining was used to quantify the number of osteoblasts in the experiment (Figures 2(a) and 2(b)). The results showed that the number of osteoblasts on the surface of bone trabeculae was reduced in high-fat diet mice and that Ferrostatin-1 inhibited the reduction in their number, since the metabolic balance of bone is maintained by a balance between osteoclast formation and bone resorption. For this reason, bone tissue was experimentally stained with TRAP (Figures 2(a) and 2(c)) to assess changes in osteoclast activity in the bone marrow cavity of mice on a high-fat diet. However, we observed no significant difference in the number of TRAP^+^ cells in the bone of mice given a high-fat diet. Therefore, these results suggest that a high-fat diet may primarily induce the loss of osteoblasts in mice.

### 3.3. Ferroptosis Plays an Important Role in High-Fat Diet-Induced Bone Loss

In previous studies, researchers found that Gpx4, a key protein for ferroptosis, is significantly altered in a high-fat environment. Immunofluorescent staining of bone tissue from mice on a high-fat diet suggested that Gpx4 protein expression was decreased in the bone marrow lumen and that this process could be reversed by Ferrostatin-1 (Figure 3(a)). The tibial bone tissues of mice were also subjected to the determination of biochemical indicators of ferroptosis, namely, total GSH, GSH/GSSG ratio, MDA, and Fe2+ content. The results showed that these MDA and Fe2+ were significantly elevated in the bone tissues of mice on a high-fat diet. However, total GSH and GSH/GSSG ratios were significantly lower. These data suggest that ferroptosis plays an important role in the high-fat diet-induced bone loss.

### 3.4. Ferroptosis Is an Important Way in Which Mc3t3-E1 Cells Undergo Death

Years of research have shown that osteogenic differentiation of Mc3t3-E1 cells is important for bone formation. If ferroptosis of Mc3t3-E1 cells is increased in a high-fat environment, its function and proliferative capacity will be greatly affected. To determine whether Mc3t3-E1 undergoes ferroptosis under high-fat conditions, immunofluorescence staining for Gpx4 and Slc7a11, the key proteins of ferroptosis, and biochemical indicators of ferroptosis, was performed. The results revealed that total GSH and total GSH/GSSG ratio were lower in Mc3t3-E1 cells treated with high-fat medium compared to the control (Figures 4(e) and 4(f)), while Fe2+ and MDA were higher in Mc3t3-E1 treated with high-fat medium (Figures 4(d) and 4(g)) and increased, and Gpx4 and Slc7a11 proteins were significantly reduced compared to the control. Moreover, the proliferation function of Mc3t3-E1 cells was somewhat restricted compared to the control group. This process could be inhibited by Ferrostatin-1. These results suggest that ferroptosis is present in Mc3t3-E1 cells cultured in a high-fat environment.

### 3.5. High-Fat Environment Inhibits Osteogenic Differentiation of Mc3t3-E1 Cells

Although cell death is an important factor affecting changes in bone mass in mice, impaired osteogenic differentiation of Mc3t3-E1 cells has a major impact on reduced bone mass in mice. Therefore, the osteogenic differentiation capacity of Mc3t3-E1 cells was examined in this experiment. During osteogenic differentiation of the cells, we found that the early marker of osteogenic differentiation, ALP, in Mc3t3-E1 cells treated with high-fat medium was significantly decreased at the seventh day of osteogenic differentiation induction (Figures 5(a) and 5(b)). The osteogenic-related proteins Osterix, Osteocalcin, and Rux2 were also reduced to varying degrees (Figures 5(c)–5(e)). And this process could be inhibited by Ferrostatin-1.

## 4. Discussion

Chronic obesity caused by a high-calorie diet has a significant negative impact on human bone mineral density (BMD) [25]. The long-term reduction in BMD and consequently osteoporosis increases the economic burden on society [26]. However, the exact mechanism of bone loss caused by a high-fat diet is not known [25]. Therefore, the search for the exact mechanism of bone loss caused by a high-calorie diet is of great importance for the prevention and treatment of bone loss. The essence of cellular ferroptosis is that lipid peroxidation and reduced expression of the core proteins Gpx4 and Slc7a11 occur in response to external stimuli that impair the cellular antioxidant system, which also affects the metabolism of cystine transport [27, 28]. In previous studies, the link between the occurrence of cellular ferroptosis and abnormal cellular function in a high-fat environment has been inextricably linked. The association between high-fat environments and cellular ferroptosis is mainly related to cardiovascular aspects [29], such as arterial lipid deposition leading to plaque formation [30], cardiac ejection capacity [31], and remodelling [32], but the mechanisms are underlying alcoholic liver disease [33]. From these studies, we can suggest that there is a link between a high-fat diet and the development of cellular ferroptosis. Therefore, it is reasonable to assume that the phenomenon of cellular ferroptosis plays an important role in the loss of bone mass in mice on a high-fat diet. In a high-fat environment, most cells undergo accumulation of lipids and excessive accumulation of reactive oxygen species [34, 35]. These are necessary conditions for ferroptosis to occur. Therefore, inhibition of ferroptosis is important in the process of impaired cellular function caused by high-fat environments. In the present experiment, mice on a high-fat diet injected with Ferrostatin-1, a ferroptosis inhibitor, showed a significant reduction in bone loss (Figure 1). In vivo experiments have confirmed the important role of ferroptosis in bone loss due to a high-fat diet. In the present study, the high-fat diet led to bone loss in mice mainly due to a disruption of the balance between osteogenesis and osteolysis, with a low number of osteoblasts, resulting in impaired osteogenic mineralization and reduced bone formation (Figure 5). In the present study, we first demonstrated in vivo experiments in animals that ferroptosis is an important influence on bone loss due to a high-fat diet. Following in vivo experiments, we found that impaired bone anabolism was an important factor in the high-fat diet-induced bone loss. The biochemical parameters of ferroptosis in mouse bone tissues also confirmed that ferroptosis occurs in the process of bone loss due to high-fat diet (Figure 3). Since osteogenic differentiation of osteoblasts is the cell that most directly affects bone synthesis, in the next study, we used in vitro culture of osteoblasts (Mc3t3-E1 cells) to verify whether bone formation of osteoblasts is affected to some extent in a high-fat environment and that cellular ferroptosis is an important factor affecting osteogenic differentiation of osteoblasts in a high-fat environment. The results of the cellular assays suggest that the high-fat environment does indeed diminish osteoblast proliferation (Figure 4) and osteogenic differentiation (Figure 5) and that this process can be mitigated by ferroptosis inhibitors. The results of this in vitro experiment are consistent with those of the in vivo experiments. It confirms that ferroptosis does occur in the high-fat environment and attenuates the normal physiological functions of the cells. The results of this study may provide a possible treatment for the reduction in bone mineral density caused by a high-fat diet. However, there are several shortcomings in this study. Firstly, a high-fat diet does not only affect the growth and development of bones but also other important organs to varying degrees. Whether damage to other important organs may indirectly lead to bone loss was also not investigated in this study. For example, it has been established that lipid deposition due to a high-fat diet has an adverse effect on blood vessels throughout the body and that the H-vessel, which represents bone anabolism, may also be significantly reduced, thereby reducing the supply of nutrients to the femoral epiphysis and indirectly leading to bone loss. Secondly, other cells that represent bone anabolism were not targeted and analyzed in this experiment, such as whether the number and function of bone marrow mesenchymal stem cells, which have the potential for multidirectional differentiation, were affected in some way and thus were a factor in bone loss in mice on a high-fat diet. In future studies, we will explore the clinical translation of cellular ferroptosis in bone loss due to high-fat diet in an effort to investigate the underlying mechanisms.

## 5. Conclusions

In the present experiment, we found that long-term high-fat diet intake led to bone loss in mice by feeding them a high-fat diet (a). And cellular ferroptosis was involved in the whole process. The results suggest that impaired bone anabolism is an important factor in bone loss in mice fed a high-fat diet (b). The reduced osteoblast differentiation function under high-fat conditions is a major factor affecting bone formation. Previous studies have found that high body weight due to high calories is an important factor contributing to bone loss in people. As people's standard of living has now improved and their diet has changed, long-term high calorie intake can lead to damage to bone microstructure. Therefore, the high-fat diet found in this experiment interferes with normal bone anabolic metabolism through the ferroptosis pathway has some clinical significance. The possible pathways by which a high-fat diet leads to bone loss are described from a mechanistic perspective. The antagonism of ferroptosis through the administration of antioxidant drugs to slow down bone loss due to high-fat diet may also be a potential clinical treatment for bone loss due to high-fat diet.

## Figures and Tables

**Figure 1:** In this experiment, it was found that feeding mice a high-fat diet reduced bone mass production and that intraperitoneal administration of the ferroptosis inhibitor Ferrostatin-1 to mice fed a high-fat diet significantly reduced the bone mass loss in mice fed a high-fat diet. Representative micro-CT images of the distal femur of mice fed a normal diet, a high-fat diet, and a high-fat diet plus a ferroptosis inhibitor for 12 weeks (a). The femoral microstructure of mice was then quantified in terms of trabecular volume fraction (BV/TV) (b), trabecular number (Tb.N) (c), trabecular thickness (Tb.Sp) (d), and trabecular separation (Tb.Th) (e). *n* = 5/group, ^∗^*P* < 0.05, ^∗∗^*P* < 0.01, ^∗∗∗^*P* < 0.001.

**Figure 2:** Chemical staining of mouse femurs with hematoxylin and eosin (H&E) after 12 weeks of feeding mice on normal and high-fat diets revealed a significant reduction in the number of metaphyseal trabeculae in the femur, which was then restored to some extent after administration of ferroptosis inhibitors (a); scale bar represents 200 *μ*m. Experiments revealed that after mice consumed a diet high in fat content, the number of alkaline phosphatase- (ALP-) positive osteoblasts on the surface of the trabeculae in the femur was significantly reduced (b), and the reduction in the number of osteoblasts was somewhat mitigated by a high-fat diet accompanied by treatment with ferroptosis inhibitors in mice. Osteoblasts are shown in brown and nuclei in green. Quantification of the number of osteoblasts per bone surface (b). Scale bars represent 100 *μ*m, *n* = 5/group, ^∗^*P* < 0.05, ^∗∗∗^*P* < 0.001. Quantification of staining for TRAP+ cells in the femoral bone marrow cavity (a, c), with osteoclasts in red and nuclei in green (a) and NS indicating no statistical difference in component; scale bars represent 100 *μ*m, *n* = 5/groups.

**Figure 3:** To demonstrate whether ferroptosis occurred in bone tissue of mice fed a high-fat diet, the expression of Gpx4 protein, a key protein for ferroptosis, in the femur of mice was examined using immunofluorescence staining. A significant decrease in the number of Gpx4 positive cells in the bone marrow of mice fed a high-fat diet was found (a), and after administration of a ferroptosis inhibitor, the number of Gpx4-positive cells increased significantly compared to the group fed a high-fat diet alone (a, b). Gpx4-positive cells in red and DAPI-stained nuclei in blue. *n* = 5/group, ^∗^*P* < 0.05, ^∗∗^*P* < 0.01. By measuring biochemical indicators of ferroptosis in the normal diet group, high-fat diet group, and high-fat diet plus ferroptosis inhibitor group, iron content (c), the total GSH content (d), GSH/GSSG ratio (e), and MDA content (f) in the femurs of mice were found to be *n* = 5/group, ^∗^*P* < 0.05, ^∗∗^*P* < 0.01; NS indicates no statistical difference.

**Figure 4:** Mc3t3-E1 cells were used as cells for the in vitro study. Mc3t3-E1 cells were treated with high-fat medium for 24 hours, and Fer-1 at a concentration of 5 *μ*mol/l was used to slow down the process of ferroptosis. 24 hours later, changes in the key ferroptosis proteins Gpx4 and Slc7a11 were measured (a, b), while there was also a significant decrease in cell proliferation capacity (c), a process that could be rescued by ferroptosis inhibitors. Some of the treated cells were also used to assay ferroptosis biochemical parameters, and intracellular iron (d), total GSH (e), GSH/GSSG (f), and MDA (g) were found to vary in the high-fat medium. *n* = 3/group, ^∗^*P* < 0.05, ^∗∗^*P* < 0.01, ^∗∗∗^*P* < 0.001.

**Figure 5:** To verify that osteogenic formation is affected to some extent in a high-fat environment. We treated Mc3t3-E1 cells in high-fat medium and then replaced the osteogenic induction medium for seven days of osteogenic differentiation culture. We found that the level of alkaline phosphatase ALP was significantly reduced in high-fat conditioned medium-treated cells at day seven of osteogenic induction culture (a, b) and that this process could be alleviated by ferroptosis inhibitors. *n* = 3/group, ^∗^*P* < 0.05, ^∗∗^*P* < 0.01. Early intracellular osteogenic differentiation was measured by immunofluorescence at day seven of osteogenic differentiation in high-fat-treated cells Osterix (c), Rux2 (d), and Ocn (e) found to be reduced to varying degrees. The addition of Fer-1, a ferroptosis inhibitor, to the high-fat medium treatment significantly reduced the expression of osteogenic marker proteins (c–e).

## Data Availability

The data that support the findings of this study are available from the corresponding author upon reasonable request.
